The article "Up-regulation of microRNA-340 promotes osteosarcoma cell apoptosis while suppressing proliferation, migration, and invasion by inactivating the CTNNB1-mediated Notch signaling pathway" was retracted in 2020. Reasons: duplicated images; signs of a paper mill; concerns about the images.

# Up-regulation of microRNA-340 promotes osteosarcoma cell apoptosis while suppressing proliferation, migration, and invasion by inactivating the CTNNB1-mediated Notch signaling pathway

**DOI:** 10.1042/BSR20171615

**Published:** 2018-08-31

**Authors:** Bao-Long Pan, Ling Wu, Li Pan, Yu-Xi Yang, Hu-Huan Li, Yan-Juan Dai, Zi-Qian He, Ling Tan, You-Guang Huang, Zong-Wu Tong, Jun-Long Liao

**Affiliations:** 1 Department of Laboratory, People’s Hospital of Yuxi City, Yuxi 653100, P.R. China; 2 Department of Quality Control, Central Blood Station of Yuxi City, Yuxi 653100, P.R. China; 3 Tumor Markers Research Center, Tumor Institute of Yunnan Province, The Third Affiliated Hospital of Kunming Medical University, Kunming 650118, P.R. China; 4 Department of Nephrology, People’s Hospital of Yuxi City, Yuxi 653100, P.R. China; 5 Department of Rehabilitation Medicine, People’s Hospital of Yuxi City, Yuxi 653100, P.R. China

**Keywords:** CTNNB1, Invasion, MicroRNA-340, Notch signaling pathway, Osteosarcoma, Proliferation

## Abstract

Osteosarcoma (OS) is the most common histological form of primary bone cancer. It is most prevalent in teenagers and young adults. The present study aims at exploring the regulatory effect of microRNA-340 (miR-340) on OS cell proliferation, invasion, migration, and apoptosis via regulating the Notch signaling pathway by targeting β-catenin (cadherin-associated protein) 1 (CTNNB1). OS tissues belonging to 45 patients and normal femoral head tissues of 45 amputees were selected. Cells were allocated to different groups. *In situ* hybridization was performed to determine the positive rate of miR-340 expression while immunohistochemistry was used to determine that of CTNNB1 and B-cell lymphoma 2 (Bcl-2). We used a series of experiments to measure the expressions of related factors and assess rates of cell proliferation, migration, invasion, cycle, and apoptosis respectively. Our results show that miR-340 was expressed a higher level in normal tissue than OS tissue. Expression of Notch, CTNNB1, hairy and enhancer of split 1 (Hes1), Bcl-2, Runt-related transcription factor 2 (Runx2), and osteocalcin increased and that of miR-340, Bcl-2 interacting mediator of cell death (BIM), and Bcl-2 associated protein X (Bax) decreased in OS tissues. U-2OS cell line had the highest miR-340 expression. We also found that the up-regulation of miR-340 had increased expression of miR-340, BIM, and Bax but decreased expression of Notch, CTNNB1, Hes1, Bcl-2, Runx2, and osteocalcin. Up-regulation of miR-340p lead to increased cell apoptosis, suppressed cell proliferation, migration, and invasion. Our study demonstrates that overexpression of miR-340 could suppress OS cell proliferation, migration, and invasion as well as promoting OS cell apoptosis by inactivating the Notch signaling pathway via down-regulating CTNNB1. Functional miR-340 overexpression might be a future therapeutic strategy for OS.

## Introduction

Osteosarcoma (OS) is a malignant primary bone tumor that affects the long bones and other bones in the whole body. It is a disease that is associated with high morbidity. OS is an aggressive neoplasm that arises from cells belonging to mesenchymal origin, which exhibits osteoblastic differentiation and produces malignant osteoid [1]. Thereinto, 78% of OS occurs in the lower extremity, 64% occurs around the knee, and 10% in the humerus [2,3]. As the most common primary bone malignancy, OS accounts for 60% of malignant childhood bone tumors but with a 60–70% survival rate of patients without metastatic diseases and less than 30% for those with OS metastasis [4]. The osteoblastic type is the predominant cell type in OS, which occupies 50–80% of OS cells with a varying fibroblastic–fibrohistiocytic or chondroblastic parts [5]. Molecular genetic abnormalities that may serve as specific markers of OS still remain unclear and the inherited cancer syndromes such as Li-Fraumeni syndrome have been reported to have association with OS [6]. Symptoms of OS include pain, swelling, limp as well as pathological fracture [7]. Chemotherapy with advanced surgery is a common approach used to treat patients with OS along with the combination of drugs such as doxorubicine and cisplatin with or without high-dose methotrexate, ifosfamide, and etoposide [3]. Despite the advances in treatment regimens, large proportions of patients with OS respond poorly to chemotherapy and have high risks of relapse or metastasis which warrant that the need for new biomarkers is discovered to help diagnose and treat patients [8].

Dysfunction of microRNAs (miRNAs) has been revealed to be associated with cancer as tumor suppressors or oncogenes by participating in biological processes like proliferation, differentiation, and apoptosis [9]. To this day, several miRNAs have been implicated in the development and progression of OS, such as miR-143, miR-199a-3p, miR-125b, miR-20a, and miR-34a. In a recent array-based screening of the potential miRNAs involved in the pathogenesis of OS, miR-340 was identified as one of 23 down-regulated miRNAs in OS samples compared with control bone [10]. However, the specific roles and underlying mechanisms of miR-340 in OS have yet to be determined. miR-340 has been verified as a tumor inhibitor in numerous human cancers that include colorectal cancer, breast cancer, gastric cancer, and OS [10–14]. Zhou et al. [10] have investigated the relationship between miR-340 and ROCK1 as well as their effects on OS cell growth, metastasis, prognosis, and progression which have led to the decision to investigating the relationship between miR-340 and OS in this present study. β-Catenin (cadherin-associated protein) 1 (CTNNB1) is a component of the cellular adhesion complexes, which links cytoplasmic tails of cadherins to α-catenin [15]. CTNNB1 regulates and coordinates cell-to-cell adhesion and gene transcription [16,17]. Mutations and overexpression of β-catenin are associated with many cancers, including hepatocellular carcinoma, colorectal carcinoma, lung cancer, malignant breast tumors, ovarian, and endometrial cancer [18]. As one of the integral structural components of cadherin-based adherens junction and the crucial nuclear effector of the canonical is the Wnt signaling pathway, the imbalance of CTNNB1 is usually related to a wide variety of diseases and dysregulated overexpression which is associated with cancers and metastasis [19]. As to patients with desmoid-type fibromatosis, overexpression of CTNNB1 has been identified to play a part in reduced event-free survival [20]. Notch is a cell surface receptor transducing short-range signals through association with transmembrane ligands on neighboring cells, and the Notch signaling pathway can regulate cell proliferation, apoptosis, and differentiation [21]. Because of its crucial role in cellular processes, effects of the Notch signaling pathway have widely been investigated in various cancers such as breast cancer, gastric cancer, and pancreatic cancer [22–24]. Due to the well-understood relation between miR-340 and OS, as well as those between CTNNB1, the Notch signaling pathway and cell biological processes, we conduct the present study in hopes of finding a theoretical foundation which will further improve our understanding of OS cells and search for new molecules for targeted therapy.

## Materials and methods

### Study subjects selection

Between March 2014 and June 2016, OS tissue samples were resected and collected from 45 patients who were pathologically diagnosed with OS in the Department of Bone Tumor of the Third Affiliated Hospital of Kunming Medical University. The exclusion criteria were as follows: (1) patients who were diagnosed with other tumors other than OS; (2) patients who have undergone radiotherapy or chemotherapy treatment; (3) patients had received other forms of anticancer therapy. Various degrees of bone destruction, soft tissue mass, and osteolytic destruction were detected using X-ray test. Within all patients, 31 were male and 14 were female ranging from 6 to 17 years old with a mean age of 8–9 years old. Next, 45 samples of normal bone tissues were collected from patients with normal femoral head tissue without a significant difference in gender and age compared with OS patients. Samples were numbered and registered after resection. Parts of the samples were used to prepare paraffin sections and the rest were stored in liquid nitrogen at −80°C. The application and use of samples were understood and approved by patients and their families. The present study was reviewed and approved by the Ethics Committee of the Third Affiliated Hospital of Kunming Medical University.

### *In situ* hybridization

Specimens were fixed in 10% formaldehyde, embedded by paraffin, and cut into 3 μm sections. Sections were transferred onto a special glass slide that was pretreated with 10% polylysine. The protocol was carried out in accordance with the manufacturer’s instructions of *in situ* hybridization kit (Boster Biological Technology Co., Ltd., Wuhan, Hubei, China). After digoxin-labeled miR-340 probe (Exiqon, Denmark) was dripped in, sections were hybridized at a constant temperature of 52°C for 16 h and then left in a warm-bath with biotinylated mouse anti-digoxin antibody at 37°C for 60 min followed by incubation in strept avidin–biotin complex (SABC). Next, diaminobenzidine (DAB) was utilized to develop color. The results were scored by two pathologists independently. Cells with blue-stained cytoplasm were considered positive. Five fields were randomly selected from each section under a light microscope (200×). Through observation, the percentage of positive cells was calculated. Specimens were considered negative if the percentage of positive cells was less than 5% and positive if the percentage was more than or equal to 5%.

### Immunohistochemistry

Specimens were dissolved in 10% neutral formalin with disodium ethylenediaminetetraacetic acid, with the pH of 7.3 and a temperature of 4°C, and the liquid was replaced every day, with approximately 6 days in total. The fixed bone tissues were rinsed with distilled water for three times, and then dehydrated it with gradient alcohol (70, 80, 95, and 100%) twice respectively. The sections were cleared with xylene I and II for 35 min, respectively, and the cleared bone tissues were immersed in paraffin wax for 3 h. Subsequently, they were embedded by paraffin and cut into 4 μm sections. Sections were dried in an incubator at 60°C for 1 h, dewaxed after drying by three cylinders of xylene for 30 min (10 min each). They were then dehydrated in three cylinders of gradient ethanol with concentration of 95, 80, and 70% respectively (1 min each). After washing with running water for 1 min, sections were incubated at 37°C with 3% H_2_O_2_ for 30 min, washed by phosphate buffer saline (PBS), and boiled in 0.01 M citrate buffer at 95°C for 20 min. After cooling to room temperature, sections were washed by PBS and sealed in normal goat serum at 37°C for 10 min. Sections were then incubated with the following primary antibodies: the rabbit polyclonal CTNNB1 (ab32572, 1:40, Abcam, Cambridge, MA, U.S.A.) and B-cell lymphoma-2 (Bcl-2, ab227801, 1:500, Abcam, Cambridge, MA, U.S.A.) at 4°C overnight followed by PBS washing for 2 min. Specimens were incubated next with horseradish peroxidase (HRP)-labeled streptavidin-working solution at 37°C for 30 min followed by PBS washing three times (5 min each time) before development by DAB (7411-49-6, Suzhou Yacoo Chemical Reagent Co., Ltd., Suzhou, Jiangsu, China). Hematoxylin (Shanghai Bogoo Biological Technological Co., Ltd., Shanghai, China) was used to restain the sections before sealing them. The positive comparison film provided by Abcam (Cambridge, MA, U.S.A.) was used as the positive control. PBS was used as the negative control, which replaced the primary antibody. Ten random fields under a high power light microscope was randomly selected from each section and used to count the percentage of positive cells with 100 cells in each field. The percentage of positive cells in the whole section ≥10% was recorded as positive and <10% as negative [25].

### Reverse transcription quantitative polymerase chain reaction (RT-qPCR)

The total RNA of tissues (the normal bone tissues were flattened with a vice, added with liquid nitrogen, and was used after grinding into powder in a mortar) and cells was extracted using the miRNeasy Mini Kit (217004, Qiagen, Hilden, Germany). The primers of miR-340, Notch, CTNNB1, Bcl-2 associated protein X (Bax), Bcl-2, Bcl-2 interacting mediator of cell death (BIM), hairy and enhancer of split 1 (Hes1), Runt-related transcription factor 2 (Runx2), and osteocalcin were designed and synthesized by Takara (Dalian, Liaoning, China) (Table 1). According to the PrimeScript RT reagent kit (Takara, Dalian, Liaoning, China), RNA was reversely transcribed to cDNA. The reverse transcription system was 10 µl. According to the instructions, the reaction conditions were set according to the following protocol: reverse transcription at 37°C for 15 min, three times, reverse transcriptase inactivation at 85°C for 5 s. The reaction mixture was selected for fluorescent quantitation PCR based on the instructions provided by the SYBR® Premix Ex Taq™ II reagent kit (Takara, Dalian, Liaoning, China). The 50 μl of reaction system consisted of 25 μl of SYBR® Premix Ex Taq^™^ II (2×), 2 μl of forward primers, 2 μl of reverse primers, 1 μl of ROX Reference dye (50×), 4 μl of DNA template, and 16 μl of ddH_2_O. RT-qPCR (7500, Applied Biosystems Inc. Carlsbad, CA, U.S.A.) was performed under the following reaction conditions: predenaturation at 95°C for 30 s, and 40 cycles of denaturation at 95°C for 5 s, annealing and extension at 60°C for 30 s. U6 was used as the internal reference for miR-340 and glyceraldehyde-3-phosphate dehydrogenase (GAPDH) was used as the reference for Notch, CTNNB1, Bax, Bcl-2, BIM, Hes1, Runx2, and osteocalcin. The mRNA relative transcriptional levels of Notch, CTNNB1, Bax, Bcl-2, BIM, Hes1, Runx2, and osteocalcin were calculated by the relative quantitative method 2^−ΔΔ*C*^_t_ with the formula: ΔΔ*C*_t_ = Δ*C*_t__(experimental group)_ − Δ*C*_t__(normal group)_, Δ*C*_t_ = *C*_t__(target gene)_ − *C*_t__(internal reference)_, and 2^−ΔΔ*C*^_t_ represented the mRNA relative transcriptional level [26].

**Table 1:** Primer sequences of genes

Genes	Sequences
MiR-340	F: 5′-ACACTCCAGCTGGGTTGGCAATGGTTAGA-3′
	R: 5′-CTCAATCGGTGTCGTGGAGTCGGCAGTTA-3′
Notch	F: 5′-GTGACTGCTCCCTCAACTTCAAT-3′
	R: 5′-CTGTCACAGTGGCCGTCACT-3′
CTNNB1	F: 5′-ACCACCAAGACTACAAGAAGCGA-3′
	R: 5′-GGATGATTTACAGGTCAGTATCGA-3′
Hes1	F: 5′-AGGCGGACATTCTGGAAATG-3′
	R: 5′-CGGTACTTCCCCAGCACACTT-3′
Runx2	F: 5′-GGCCCAGTGGCATGGTCGACACATCCCGCATGTG-3′
	R: 5′-CACATGCGGGATGTGTCGACCATGCCACTGGGCC-3′
Osteocalcin	F: 5′-GTCACGCGTAGAAGCTTGGTACCAGGA-3′
	R: 5′-GGCCTCGAGCGGCAGCCTCCAGCACTG-3′
BIM	F: 5′-CGTAGCGCATGCGATA-3′
	R: 5′-CATGCCGTATAAGCTAGTT-3′
Bax	F: 5′-GGCCCACCAGCTCTGAGCAGA-3′
	R: 5′-GCCACGTGGGGGTCCCAAAGT-3′
Bcl-2	F: 5′-TTTGAGTTCGGTGGGGTCATC-3′
	R: 5′-CCAGGAGAAATCAAACAGAGG-3′
U6	F: 5′- CTCGCTTCGGCAGCACA-3′
	R: 5′-AACGCTTCACGAATTTGCGT-3′
GAPDH	F: 5′-TGCACCACCAACTGCTTAGC-3′
	R: 5′- GGCATGGACTGTGGTCATGAG-3′

Abbreviations: Bax, Bcl-2 associated protein X; BIM, Bcl-2 interacting mediator of cell death; CTNNB1, β-catenin (cadherin-associated protein) 1; F, forward; GAPDH, glyceraldehyde-3-phosphate dehydrogenase; Hes1, hairy and enhancer of split 1; miR-340, microRNA-340; R, reverse; Runx2, Runt-related transcription factor 2.

### Western blot analysis

Protein of tissues and cells was extracted using a RIPA lysis buffer kit (R0010, Solarbio, Beijing, China). Protein concentration was measured by the bicinchoninic acid (BCA) method (69-21875, MSK Biological Technological Co., Ltd., Wuhan, China). After 10% sodium dodecyl sulfate-polyacrylamide gel electrophoresis (SDS-PAGE, 20050227, Beyotime Biotechnology, Haimen, Jiangsu, China), the membrane was transferred and underwent antigen-antibody reaction. Primary antibodies including Notch antibody (1:75, ab27526), CTNNB1 antibody (1:5000, ab32572), Hes1 antibody (1:50, ab71559), BIM antibody (1:2000, ab32158), Bax antibody (1:2000, ab32503), Bcl-2 antibody (1:2000, ab32124), Runx2 antibody (1:10000, ab76956), osteocalcin antibody (1:10000, ab19857), and GAPDH antibody (1:1000, ab9485) which were purchased from Abcam (Cambridge, MA, USA) were added to the membrane and incubated at 4°C overnight. The membrane was then incubated with HRP-labeled goat-anti-rabbit IgG secondary antibody (1:1000, BA1056, BOSTER Biological Technology Co., Ltd., Wuhan, Hubei, China) and then immersed in electrochemiluminescence (ECL, WBKLS0500, Pierce, Rockford., IL, U.S.A.). The result was observed after developing the color in a dark room and photographs were taken. GAPDH was used as the internal protein reference and the relative protein expression level was presented as the gray value ratio of target band to the internal reference band.

### Dual-luciferase reporter assay

Luciferase reporter assay was performed to verify whether CTNNB1 was the direct target of miR-340. The restriction site Spe I and Hind III were used to introduce artificially synthesized gene segments of CTNNB1′UTR to pMIR-reporter. Mutant sites of complementary sequences of seed sequences were designed on the CTNNB1 wild-type (WT) (forward primer sequence: 5′-ACCACCAAGACTACAAGAAGCGA-3′; reverse primer sequence: 5′-GGATGATTTACAGGTCAGTATCGA-3′). After restriction enzyme digestion, target segments were inserted into pMIR-reporter plasmid using T4 DNA ligase.

The correct luciferase reporter plasmids of WT and mutant type (MUT) were cotransfected into HEK-293T cells (Shanghai Beinuo Biological Technology Co. Ltd., Shanghai, China) with miR-340 respectively. Cells were harvested and lysed 48 h after transfection, and luciferase activity was measured using a dual-luciferase reporter assay kit.

### Cell culture, grouping, and transfection

SOSP-9607, U-2OS, and MG63 cell lines purchased from the Shanghai Cell Centre (Shanghai, China) were inoculated in cell culture medium and cultured at 37°C in an incubator with 5% CO_2_. The medium was composed of 10% fetal bovine serum (FBS), RPMI-1640 medium and mycillin, and was replaced every 24–48 h. Cells were treated and digested with 0.25% trypsin and then passaged. Cells of the third generation were selected and collected for further experiments. RT-qPCR was performed to determine miR-340 expression in each cell line and the cell line with the highest relative expression was selected for subsequent experiments. Cells were assigned into the following six groups: blank, NC, miR-340 mimic, miR-340 inhibitor, siRNA-CTNNB1 and miR-340 inhibitor + siRNA-CTNNB1. All cells were seeded in a six-well plate 24 h before transfection. When cell confluence reached 50%, cells were transfected with human OS cell lines under the mediation of liposome lipofectamine2000 (11668027, Invitrogen, Carlsbad, CA, U.S.A.). A total of 100 pmoL blank, NC, miR-340 mimic, miR-340 inhibitor, siRNA-CTNNB1, and miR-340 inhibitor + siRNA-CTNNB1 were diluted by 250 µl of serum-free Opti-MEM medium (31985-070, Gibco, Carlsbad, CA, U.S.A.) (the final concentration added to cells was 50 nM), gently mixed, and incubated at room temperature for 5 min. Two hundred and fifty microliters of serum-free Opti-MEM medium was then used to dilute 5 µl of lipofectamin 2000 and lightly mixed followed by incubation at room temperature for 5 min. The mixed aforementioned two solutions were incubated at room temperature for 20 min, and added into corresponding cell culture plates. After incubation at 37°C in an incubator with 5% CO_2_ for 6–8 h, the medium was replaced with a new complete medium. After incubation for another 24–48 h, subsequent experiments were performed on cells obtained from the culture.

### 3-(4,5-dimethylthiazol-2-yl)-2,5-diphenyltetrazolium bromide (MTT) assay

When the cell density in each group reached 80%, cells were washed with PBS twice, treated with conventional trypsin with single-cell suspension produced using a straw. A cell counter (Beckman Coulter, Inc., Fullerton, CA, U.S.A.) was applied too for cell counting. Then, cells were cultured in a 96-well plate (200 μl/well) with six duplicated wells with 3–6 × 10^3^ cells per well. The cultured cells were incubated at 37°C in an incubator with 5% CO_2_ for 24–72 h and supplemented with 20 μl of MTT solution (5 mg/ml, Sigma, St. Louis, MO, U.S.A.) to develop the color. Cells were further incubated at 37°C in an incubator with 5% CO_2_ for another 4 h and the nutrient solution was removed when the culture was terminated. Subsequently, 150 μl of dimethylsulfoxide (DMSO) (Beijing Chemical Works, Beijing, China) was added into each well and lightly shaken for 10 min to allow the formazan crystals produced by living cells to dissolve. The optical density (OD) value at the wavelength of 490 nm after 24, 48 and 72 h were measured respectively using an enzyme-linked immunometric meter (mode 680, Bio-Rad, Hercules, CA, U.S.A.). The cell viability curve was produced by plotting the time point as the *X*-axis and the OD value as *Y*-axis. Each experiment was repeated three times.

### Flow cytometry

Propidium iodide (PI) was applied to determine cell cycle. The collected cells were fixed in 70% ice ethanol and incubated at 4°C overnight. Cells were centrifuged at 800×***g*** with the supernatant removed afterward, followed by PBS rinse containing 1% FBS twice. Cells were resuspended in 400 μl of binding buffer followed by the addition of 50 μl of RNA enzyme a (Sigma, St. Louis, MO, U.S.A.) and left to incubate at 37°C for 30 min. Fifty microliters of 50 mg/l PI (Sigma, St. Louis, MO, U.S.A.) was added to the cells and left to incubate in the dark at room temperature. A flow cytometer system was used to determine the cell cycle of the samples.

Cell apoptosis was detected by Annexin-V-fluorescein isothiocyanate (FITC)/PI double staining. OS cells were seeded in a six-well plate (2 × 10^5^ cells/well) and transfected respectively with 100 nmol/l. The solution was removed 72 h after transfection and cells were washed by 4°C precooled PBS and digested by trypsin. Cells were transferred to a 15 ml of centrifuging tube, and centrifuged at 800×***g*** with the supernatant removed afterward. The precipitate was then washed with PBS twice. According to the instructions provided by the Annexin-V-FITC apoptosis detection kit I (556547, BD Biosciences, San Diego, CA, U.S.A.), cells were resuspended in 500 μl of binding buffer, and mixed with 5 μl of FITC and 5 μl of PI and left to incubate at room temperature for 15 min. Finally, apoptosis was detected with flow cytometry.

### Scratch test

Cells after transfection in the six groups of the six-well plate were selected correspondingly. Horizontal lines were created evenly every 0.5–1 cm across the well on the back of each plate using a ruler by a maker pen. Each well was traversed by five lines at least, and cultured with 5 × 10^5^ cells overnight. On the next day, scratches perpendicular to the transverse line were made with the help of the ruler using a transfer liquid gun on the back of a six-well culture plate. PBS was used to wash cells three times and cells scratched out were removed. The remaining cells were cultured with serum-free medium in an incubator with 5% CO_2_ at 37°C. After that, samples were selected separately at 0, 12 and 24 h, and photographed under an inverted light microscope (×100) to measure the scratch distance.

### Transwell assay

Matrigel (50 mg/l; Sigma, St. Louis, MO, U.S.A.) was diluted at the ratio of 1:8 and 60 μl of diluted matrigel was added onto the surface of the upper chamber of the basement membrane. After air-drying at room temperature, the remaining liquid was removed. Serum-free solution (50 μl) containing 10 g/l albumin from bovine (BSA) was added to each well and left at 37°C for 30 min. Cells in the logarithmic growth phrase were selected and density adjusted to 1 × 10^5^ cells/ml with serum-free medium containing 10 g/l fetal bovine serum (FBS). Then, 200 μl of cell suspension was added to each transwell chamber. Approximately 500 μl of 100 ml/l FBS was added to the lower chamber of the 24-well plate and left to incubate in an incubator with 5% CO_2_ for 24 h. When the chamber was taken out, cells on the polyvinylidene fluoride (PVPF) membrane close to the inner side of chamber were wiped out using cotton buds. The chamber was fixed in 95% ethanol for 30 min, stained with Crystal Violet (Sigma, St. Louis, MO, U.S.A.) for 20 min, and washed by water three times. The cells in the chambers were observed, counted, and photographed under an inverted light microscope (Olympus, Tokyo, Japan).

### Statistical analysis

All experimental data were processed by SPSS 21.0 statistical software (IBM Corp., Armonk, NY, U.S.A.). Measurement data were expressed as a mean ± standard deviation. Comparisons between two data groups were performed by a *t*-test and comparisons made among multiple groups were analyzed by a one-way analysis of variance (ANOVA). Values of *P*<0.05 were indicative of significant statistical difference.

## Results

### miR-340 is closely related to cell invasion, cell metastasis, and enneking staging of OS

Initially, *in situ* hybridization was performed to measure the expression levels of miR-340 and to investigate the correlation between miR-340 and clinicopathological features in normal and OS tissues. The results showed that miR-340 was mainly expressed in the cytoplasm. Positive cells were presented as tan-colored particles while positive rate of miR-340 was significantly lower in OS tissue than that of normal tissues (*P*<0.05) (Figure 1A,B). The correlation between miR-340 and clinicopathological features revealed that miR-340 expression was closely related to invasion, metastasis, and enneking staging of patients with OS. In comparison with specimens without invasion and metastasis, specimens with invasion and metastasis had lower miR-340 positive rate (*P*<0.05). Moreover, the positive rates of miR-340 expression showed an increase from enneking stage III, II to I (*P*<0.05). However, no correlations were found between the gender or age of patients with tumor size (*P*>0.05) (Table 2).

**Figure 1:** Positive expression rates of miR-340 in OS and normal bone tissues detected by *in situ* hybridization (**A**) *In situ* hybridization images (×200) of normal bone and OS tissues. (**B**) Positive expression rate of miR-340 in normal bone and OS tissues; *P<0.05 vs*.* the normal group; miR-340, microRNA-340; OS, osteosarcoma.

**Table 2:** Correlation between miR-340 and clinicopathological features of OS

Clinicopathological features	*n*	miR-340		Positive rate (%)	*P*
		+	-		
Age (years)					
<15	15	6	9	40.00%	>0.05
≥15	30	13	17	43.33%	
Gender					
Male	31	17	16	54.84%	>0.05
Female	14	8	6	57.14%	
Tumor diameter					
<5 cm	21	9	12	42.86%	>0.05
≥5 cm	24	11	13	45.83%	
Invasion and metastasis					
Yes	22	5	17	22.72%	<0.05
No	23	12	11	52.17%	
Enneking staging					<0.05
Stage I	14	8	6	57.14%	
Stage II	22	9	13	40.91%	
Stage III	9	2	7	22.22%	

Abbreviation: miR-340, microRNA-340.

### OS tissues had higher positive expression rate of CTNNB1 and Bcl-2

We performed immunohistochemistry analysis to identify the protein expression of CTNNB1 and Bcl-2. CTNNB1 protein was stained on the cytoplasm and was deemed positive by the appearance of yellow or brown granules in the cytoplasm. The positive rate of CTNNB1 in normal bone tissues was significantly lower than that of OS tissues (*P*<0.05) (Figure 2). Bcl-2 was mainly expressed on the membrane with the existence of yellow particles as positive. The positive rate of Bcl-2 in normal tissue was significantly lower than that in OS tissue (*P*<0.05). The results demonstrated that OS tissues had a higher positive expression rate of CTNNB1 and Bcl-2.

**Figure 2:** Immunohistochemistry and positive expression rate of CTNNB1 and Bcl-2 protein in OS and normal bone tissue (**A**) Immunohistochemical images (×200) of CTNNB1 in normal bone and OS tissues. (**B**) Positive expression rate of CTNNB1 in normal bone and OS tissues. (**C**) Immunohistochemical images (×200) of Bcl-2 in normal bone and OS tissues. (**D**) Positive expression rate of Bcl-2 in normal bone and OS tissues; *P<0.05 vs*.* the normal group; Bcl-2, B-cell lymphoma-2; CTNNB1, β-catenin (cadherin-associated protein) 1; OS, osteosarcoma.

### miR-340 is down-regulated while CTNNB1 is up-regulated in OS tissue

RT-qPCR and Western blot analysis were performed to measure miR-340 expression along with mRNA and protein expression of CTNNB1, BIM, Bax, Notch, CTNNB1, Hes1, Bcl-2, Runx2, and osteocalcin in normal and OS tissues. The results revealed compared with normal bone tissues, OS tissues exhibited lower miR-340 expression, mRNA expression and protein level of BIM and Bax but increased mRNA and protein expression of Notch, CTNNB1, Hes1, Bcl-2, Runx2, and osteocalcin (all *P*<0.05) (Figures 3 and 4). The results above indicated that miR-340 is poorly expressed while CTNNB1 is up-regulated in OS tissues.

**Figure 3:** RT-qPCR detection of miR-340 expression and relative mRNA expression of Notch, CTNNB1, Bax, Bcl-2, BIM, Hes1, Runx2, and osteocalcin in OS and normal bone tissues *P<0.05 vs*.* the normal group; Bax, Bcl-2 associated protein X; Bcl-2, B-cell lymphoma 2; BIM, Bcl-2 interacting mediator of cell death; CTNNB1, β-catenin (cadherin-associated protein) 1; Hes1, hairy and enhancer of split 1; miR-340, microRNA-340; OS, osteosarcoma; Runx2, Runt-related transcription factor 2.

**Figure 4:** Western blot analysis of the relative protein expression of Notch, CTNNB1, Bax, Bcl-2, BIM, Hes1, Runx2, and osteocalcin in OS and normal bone tissues (**A**) Relative protein expression of Notch, CTNNB1, Bax, Bcl-2, BIM, Hes1, Runx2, and osteocalcin. (**B**) Protein bands of Notch, CTNNB1, Bax, Bcl-2, BIM, Hes1, Runx2, and osteocalcin by Western blot analysis; *P<0.05 vs*.* the normal group; Bax, Bcl-2 associated protein X; Bcl-2, B-cell lymphoma 2; BIM, Bcl-2 interacting mediator of cell death; CTNNB1, β-catenin (cadherin-associated protein) 1; GAPDH, glyceraldehyde-3-phosphate dehydrogenase; Hes1, hairy and enhancer of split 1; OS, osteosarcoma; Runx2, Runt-related transcription factor 2.

### U-2OS cell line exhibited the highest miR-340 expression

RT-qPCR was carried out in order to select the cell line with the highest miR-340 expression from the following three human OS cell lines: SOSP-9607, U-2OS, and MG63. Results in Figure 5 help illustrate the different miR-340 expressions in three OS cell lines whereby U-2OS cell line exhibited the highest miR-340 expression (*P*<0.05). Therefore, the U-2OS cell line was selected for the subsequent experiments.

**Figure 5:** miR-340 expression in SOSP-9607, U-2OS, and MG63 cell lines *P<0.05 vs*.* SOSP-9607 cell line; ^#^*P*<0.05 vs*.* MG63 cell line; miR-340, microRNA-340.

### CTNNB1 is a direct target gene of miR-340

We examined whether miR-340 could directly regulate CTNNB1 by means of target prediction program and luciferase activity determination. Based on the analysis of online software, we found a specific binding region between the gene sequence of CTNNB1 and miR-340 sequence, indicating that CTNNB1 was a target gene of miR-340 (Figure 6A). We then carried out a dual-luciferase reporter assay which further verified that CTNNB1 was a target gene of miR-340 (Figure 6B). Compared with the NC group, the luciferase activity of Wt-miR-340/CTNNB1 was significantly inhibited by miR-340 (*P*<0.05) while the luciferase activity of MUT 3′URT did not exhibit the same effect (*P*>0.05). Therefore, we can conclude that miR-340 could specifically bind to CTNNB1 gene.

**Figure 6:** CTNNB1 is a direct target gene of miR-340 by means of target prediction program and luciferase activity determination *P<0.05 vs*.* the normal group. (**A**) The predicative binding site of miR-340 on CTNNB1 3′URT. (**B**) Histogram of luciferase activity; 3′URT, 3′untranslated region; CTNNB1, β-catenin (cadherin-associated protein) 1; miR-340, microRNA-340.

### Up-regulation of miR-340 functionally suppresses CTNNB1

RT-qPCR was conducted following transfection to investigate whether miR-340 could affect mRNA expressions of CTNNB1, BIM, Bax, Notch, CTNNB1, Hes1, Bcl-2, Runx2, and osteocalcin. The blank and NC groups showed no significant difference regarding above-mentioned expression levels (Figure 7) (*P*>0.05). Compared with the blank and NC groups, U-2OS cell line in the miR-340 mimic and siRNA-CTNNB1 groups had higher mRNA expression of BIX and Bax but lower mRNA expressions of CTNNB1, Notch, Bcl-2, Hes1, Runx2, and osteocalcin while the opposite trend was seen in the miR-340 inhibitor group (all *P*<0.05). On the other hand, the miR-340 mimic group had elevated miR-340 expression (*P*<0.05) while the siRNA-CTNNB1 group had no significant difference in miR-340 expression (*P*>0.05). The miR-340 inhibitor + siRNA-CTNNB1 group had significantly lower miR-340 expression (*P*<0.05) but had no significant differences in the mRNA expression of Notch, CTNNB1, Bax, Bcl-2, Hes1, BIX, Runx2, and osteocalcin (*P*>0.05). Thus, our results suggest that miR-340 might down-regulate CTNNB1.

**Figure 7:** RT-qPCR detection of miR-340 expression and relative mRNA expression of Notch, CTNNB1, Bax, Bcl-2, BIM, Hes1, Runx2, and osteocalcin in each transfected group *P<0.05 vs*.* the NC group; Bax, Bcl-2 associated protein X; Bcl-2, B-cell lymphoma 2; BIM, Bcl-2 interacting mediator of cell death; CTNNB1, β-catenin (cadherin-associated protein) 1; Hes1, hairy and enhancer of split 1; miR-340, microRNA-340; Runx2, Runt-related transcription factor 2.

A Western blot analysis was conducted to investigate whether miR-340 could alter the protein expressions of CTNNB1, BIM, Bax, Notch, CTNNB1, Hes1, Bcl-2, Runx2, and osteocalcin after transfection (Figure 8). We found no significant differences between the blank and NC groups (*P*>0.05). Compared with the blank and NC groups, the U-2OS cell line in the miR-340 mimic and siRNA-CTNNB1 groups had higher protein levels of BIX and Bax but lower protein levels of CTNNB1, Notch, Bcl-2, Hes1, Runx2, and osteocalcin while opposite trend was observed in the miR-340 inhibitor group (all *P*<0.05). We also found no significant differences in protein levels in the miR-340 inhibitor + siRNA-CTNNB1 group (*P*>0.05).

**Figure 8:** Western blot analysis of the protein expressions of Notch, CTNNB1, Bax, Bcl-2, BIM, Hes1, Runx2, and osteocalcin in each transfected group (**A**) Relative protein expression of Notch, CTNNB1, Bax, Bcl-2, BIM, Hes1, Runx2, and osteocalcin in each group. (**B**) Protein bands of Notch, CTNNB1, Bax, Bcl-2, BIM, Hes1, Runx2, and osteocalcin by Western blot analysis; *P<0.05 vs*.* the NC group; Bax, Bcl-2 associated protein X; Bcl-2, B-cell lymphoma 2; BIM, Bcl-2 interacting mediator of cell death; CTNNB1, β-catenin (cadherin-associated protein) 1; GAPDH, glyceraldehyde-3-phosphate dehydrogenase; Hes1, hairy and enhancer of split 1; miR-340, microRNA-340; NC, negative control; Runx2, Runt-related transcription factor 2.

### Up-regulation of MIR-340 or SIRNA-CTNNB1 inhibited OS cell proliferation

As depicted in Figure 9, the MTT assay revealed that the proliferation rate was significantly different at the 48 and 72 h time points compared with the 24-h time period (*P*<0.05). There were no significant differences observed in relation to cell proliferation between the blank group and the NC group (*P*>0.05). Compared with the blank and NC groups, the cell proliferation rate was lower in the miR-340 mimic and siRNA-CTNNB1 groups at 48 and 72 h after transfection but was higher in the miR-340 inhibitor group (all *P*<0.05). The miR-340 inhibitor + siRNA-CTNNB1 group had no significant difference as to cell proliferation (*P*>0.05). These findings indicated that up-regulation of miR-340 or silencing of CTNNB1 could reduce U-2OS cell proliferation *in vitro* while down-regulation of miR-340 expression could promote U-2OS cell proliferation *in vitro*.

**Figure 9:** Changes of cell proliferation in each group after transfection determined by MTT assay *P<0.05 vs*.* the blank and NC groups; CTNNB1, β-catenin (cadherin-associated protein) 1; miR-340, microRNA-340; NC, negative control; OD, optical density.

### Up-regulation of miR-340 or silencing CTNNB1 suppressed OS cell migration and invasion

A scratch test and Transwell assay was conducted to investigate the miR-340 and CTNNB1 and their respective effects on cell migration and invasion. The results of scratch test showed that the blank, NC, and miR-340 inhibitor + siRNA-CTNNB1 groups exhibited no significant differences in cell migration as did the miR-340 mimic and siRNA-CTNNB1 groups (*P*>0.05). Compared with the blank and NC groups, the miR-340 mimic and siRNA-CTNNB1 groups showed a significant decrease in cell migration (*P*<0.05) where the opposite trend was found in the miR-340 inhibitor group (*P*<0.05) (Figure 10A,C).

**Figure 10:** Scratch test and Transwell assay analysis of OS cell migration and invasion (**A**) Images (×100) of scratch test under the microscope at 0 and 24 h. (**B**) Images (×200) of Transwell assay under the microscope. (**C**) Histogram of migration distances. (**D**) Histogram of cell numbers transferred from the upper transwell chamber to the lower chamber; *P<0.05 vs*.* the blank and NC groups; CTNNB1, β-catenin (cadherin-associated protein) 1; miR-340, microRNA-340; NC, negative control.

From the results obtained by the Transwell assay, we found no significant differences among the blank, NC, and miR-340 inhibitor + siRNA-CTNNB1 groups in the amount of cells that were transferred from the upper chamber to the lower chamber (*P*>0.05). Similarly, the miR-340 mimic and siRNA-CTNNB1 groups showed no obvious difference (*P*>0.05). Compared with the blank and NC groups, the miR-340 mimic and siRNA-CTNNB1 groups had a significantly lower number of cells that were transferred from the upper chamber to the lower chamber (*P*<0.05) with opposite trend found in the miR-340 inhibitor group (*P*<0.05) (Figure 10B,D). All in all, our results indicated that overexpressed miR-340 or CTNNB1 silencing suppresses cell migration and cell invasion of OS cells.

### Up-regulation of miR-340 or silencing CTNNB1 affected cell cycle distribution and promoted cell apoptosis

Flow cytometry was applied to determine whether miR-340 and CTNNB1 could influence the cell cycle distribution as well as apoptosis. The results of PI single staining (Figure 11) showed that the blank and NC groups had no obvious difference in cell cycle distribution (*P*>0.05). Compared with the blank and NC groups, the miR-340 mimic and miR-340 inhibitor + siRNA-CTNNB1 groups had a higher proportion of cells that were arrested in G0/G1 phase and a lesser amount of cells in S phase. This indicates that OS cell proliferation was significantly suppressed whereby the opposite trend found in the miR-340 inhibitor group (all *P*<0.05). No significant differences existed among the blank, NC, and miR-340 inhibitor + siRNA-CTNNB1 groups (*P*>0.05). Thus, our results indicated that up-regulation of miR-340 or silencing CTNNB1 expression might play an important role in the cell cycle distribution of OS cells.

**Figure 11:** OS cell cycle distribution in each group after transfection by PI double staining (**A**) Chart of cell cycle in each group. (**B**) Histogram of cells in each phase in each group; *P<0.05 vs. the blank and NC groups; CTNNB1, β-catenin (cadherin-associated protein) 1; miR-340, microRNA-340; NC, negative control.

Results of Annexin-V-FITC/PI double staining are shown in Figure 12. There were no significant differences in the rates of cell apoptosis detected between the blank and NC groups (*P*>0.05). Compared with the blank and NC groups, the miR-340 inhibitor group inhibited cell apoptosis while the miR-340 mimic and siRNA-CTNNB1 groups were found to accelerate cell apoptosis (all *P*<0.05). No significant differences existed among the blank, NC, and miR-340 inhibitor + siRNA-CTNNB1 groups (*P*>0.05). The available evidence suggests that the up-regulation of miR-340 or silence of CTNNB1 could promote OS cell apoptosis.

**Figure 12:** Cell apoptosis in each group after transfection by Annexin-V-FITC/PI double staining (**A**) Diagram of cell apoptosis in each group; (**B**) Histogram of cell apoptosis rates in each group; *P<0.05 vs*.* the blank and NC groups; CTNNB1, β-catenin (cadherin-associated protein) 1; miR-340, microRNA-340; NC, negative control.

## Discussion

Inheriting from the primitive bone-forming mesenchymal cells, OS is a primary bone malignancy that mainly affects growing bones of children and adolescents and is associated with high morbidity [27]. As a result of OS’ remarkable genetic complexity, the absence of recognizable precursor lesions and insufficient knowledge of its origin, it has been hard to identify the molecular features and pathologies of OS [28]. miR-340 and OS are related to one another [29]. We have incorporated CTNNB1 and the Notch signaling pathway into the study to find a new theoretical basis for the treatment of OS. In the present study, we investigated the up-regulation of miR-340 suppressed OS cell proliferation, migration, and invasion and inducing OS cell apoptosis by negatively regulating CTNNB1 via inhibition of the Notch signaling pathway.

First, our study revealed that cells transfected with miR-340 mimics had increased expression levels of miR-340, BIM, and Bax but decreased expression of Notch, CTNNB1, Hes1, Bcl-2, Runx2, and osteocalcin. It has been reported that in endometrial carcinoma, overexpression of miR-340 leads to increased Bax protein expression and decreased Bcl-2 protein expression [30]. An antagonizing relation exists between Bcl-2 and BIM whereby BIM would be free to increase cell apoptosis by activating Bax [31]. Cancer cells develop mechanisms that suppress BIM expression, which allows for tumor progression and metastasis [32]. In nephron progenitors, the proapoptotic protein BIM has been validated as an miRNA target of miR-17–92 and miR-106a–363 where by the same expression pattern has also been noticed in miR-181a and BIM has been observed by He et al*.* [33,34]. Mutations in CTNNB1, which encodes β-catenin, have been presented in a great number of malignant and benign neoplasms [35]. Mohammadi-Yeganeh et al*.* [36] have reported increasing miR-340 in breast cancer led to significantly decreased expressions of its target genes; CTNNB1, ROCK1, and c-MYC by directly interacting with their 3′UTRs. Recently, Song et al. [37] have also verified the target regulation relationship between miR-340 and CTNNB1 and identified that cells transfected with miR-340 mimics lowered CTNNB1 expression by targeting 3′UTR of CTNNB1 mRNA. It has been demonstrated that β-catenin induced Hes1 promoter activation via β-catenin siRNA which illustrated the identical expression trends of them too [38]. Hes1 is a downstream effector of the Notch signaling pathway, which has the same trend of expression with Notch in OS [39]. Its effect on Notch has been linked to its influence on the maintenance of stem cells and progenitor cells [40]. The Notch signaling pathway in OS is also influenced by its downstream genes DTX1 and Hes1 [39]. Inhibition of both the Wnt–β-catenin and Notch signaling pathways could sensitize OS cells to chemotherapy [41]. The transcription factor Runx2 also has been found negatively regulated by miR-204 and miR-211 to inhibit osteogenesis by binding to Runx2 3′UTR [42]. Osteocalcin, as a key marker of osteoblast activity and bone formation, can not only affect osteoid mineralization but also play a part in negative feedback during the process of bone remodeling [43,44]. Positive osteocalcin exists in malignant osteoblasts in all cases of OS [45]. Identical expression trends of β-catenin, Runx2, and the most osteoblast-specific gene osteocalcin have been previously observed in osteoblastic cells [46,47]. Therefore, it is reasonable to conclude that in OS cells, overexpression of miR-340 increases the BIM and Bax expression but leads to a decrease in the expression of Notch, CTNNB1, Hes1, Bcl-2, Runx2, and osteocalcin.

We found that transfecting cells with miR-340 mimics leads to increased cell apoptosis and inhibits cell proliferation, migration, and invasion by targeting CTNNB1 via inhibition of the Notch signaling pathway. The inhibitory role of miR-340 in cell proliferation, migration, and invasion has been mentioned in various cancers such as breast cancer, colorectal cancer, melanoma, and OS [11,12,14,29,48]. A similar role of miR-340 has been documented regarding endometrial carcinoma that up-regulation of miR-340 can induce apoptosis by increasing Bax (proapoptosis) and decreasing Bcl-2 (antiapoptosis) in RL 95-2 cells which is in accordance with our aforementioned results [30]. β-Catenin, which is direct targeted by miR-340 in mesenchymal stem cells, is essential for osteogenic differentiation [49]. It has been illustrated that the Wnt signaling pathway plays a significant role in osteoblast at different levels such as proliferation and apoptosis and the realization of its functions relies mainly on the stabilization of β-catenin associating with Tcf/Lef family of transcription factors [50]. Inactivation of the Notch signaling pathway decreases OS cell proliferation and migration [51]. This was supported by data from another study that showed that activation of Notch signaling may contribute to the development of canine OS. However, association of low HES1 expression and shorter DFI suggests that mechanisms that do not alter HES1 expression may drive the most aggressive tumors [52]. By reciprocal inhibition of its downstream effectors, deltex1 and hes1, the Notch signaling pathway blocks OS invasion [39]. It has also been discussed that γ-secretase protein complex could inhibit the Notch signaling pathway to suppress cell proliferation and lead to cell apoptosis [53]. Ma et al. [41] have claimed that since γ-secretase inhibitor prevented OS cell invasion and reduced tumor growth of mouse xenografts, the Wnt–β-catenin and Notch signaling pathway inhibitor together could be applied to improve outcomes of OS treatment. Zhou et al*.* [10] have also elucidated that the overexpression of miR-340 suppressed OS cell migration, invasion, proliferation, and metastasis by down-regulating its direct target ROCK1. In line with these studies, our study demonstrated that miR-340 was able to inhibit OS cell proliferation, invasion and migration, and induce OS cell apoptosis by inactivating the Notch signaling pathway via CTNNB1 targeting.

As for the *in vivo* results, in human OS with the high molecular homology, there is a potential role of miR-133b and miR-1 as biomarkers for OS treatment in canine [54]. Additionally, it has been reported that overexpression of miR-340 significantly inhibited tumor growth and metastasis in a xenograft mouse model with OS [10]. Besides, an investigation on a potential role of miR-144 on tumorigenesis and metastasis of OS in a murine model has found that overexpression of miR-144 inhibited the metastasis of OS cells *in vivo* [55]. All these aforementioned results demonstrate that miR-340 plays a protective role in the treatment of OS.

To sum up, our study demonstrated that miR-340 suppresses OS cell proliferation, migration, and invasion but promoted OS cell apoptosis by inactivating the Notch signaling pathway via the inhibiting CTNNB1. As mentioned above, *in vitro* studies indicated that overexpression of miR-340 protects against OS through the inactivation of the CTNNB1-mediated Notch signaling pathway, suggesting the functional miR-340 overexpression might be a future therapeutic strategy for OS. Additionally, as previously mentioned in the *in vivo* information from other studies, we draw a conclusion that miRNA, such as miR-340, is required for the protection against OS. Considering the strong miR-340-mediated tumor suppression supported by our study, together with the highly promising therapeutic approaches depend on the re-expression of tumor suppressor miRNAs, further studies are warranted, to explore the potential of miR-340 as a therapeutic tool in OS.

## Abbreviations

Bax: Bcl-2 associated protein X
Bcl-2: B-cell lymphoma 2
BIM: Bcl-2 interacting mediator of cell death
CTNNB1: β-catenin (cadherin-associated protein) 1
Hes1: hairy and enhancer of split 1
OS: osteosarcoma
Runx2: Runt-related transcription factor 2
